# An Empirical Study on the Relationship between Community Sports Activities and Community Residents' Mental Health

**DOI:** 10.1155/2022/3836758

**Published:** 2022-02-28

**Authors:** Daojun Wang, Xinli Xing

**Affiliations:** Department of Physical Education, Qingdao Agricultural University, Qingdao 266109, Shandong, China

## Abstract

A full understanding of mental health can improve people's ability to identify mental diseases and cope with psychological problems, so as to improve the ability of the whole community to resist mental diseases. Community health education is particularly important in community mental health service. The traditional health education mode is carried out through lectures or paper brochures, and the effect is not significant, so we need to constantly improve the health education mode. Through the development of community mental health education and service, we can improve people's mental health quality and promote family happiness and social stability. Based on this, this study mainly analyzes the relationship between community sports activities and mental health of community residents. Physical exercise can reduce stress reaction, regulate emotion, enhance mental health, prevent, and treat mental diseases. Therefore, physical exercise has been used not only as a method to enhance physical fitness but also as an important means to regulate psychology.

## 1. Introduction

Mental health service is an important part of community health service. It is one of the important ways to help people eliminate psychological conflicts, help residents balance their mentality, soothe psychological trauma, resolve social and family conflicts, relieve residents' various pressures and tensions, and finally enhance residents' mental health quality [1]. Physical exercise can reduce stress reaction, regulate emotion, enhance mental health, and prevent and treat mental diseases. Therefore, physical exercise has been used not only as a method to enhance physical fitness but also as an important means to regulate psychology [2]. With the reform of the health system and medical security system, community health service has become an important work of health administrative departments. From the modern development concept of mental health, improving the level of mental health can improve the efficiency of study, work, and quality of life and reduce the occurrence of various mental diseases [3]. In recent years, with the improvement of people's living standards, the demand for material life and spiritual life has been increasing. With the gradual improvement of China's socialist market economic system, the leisure time of urban residents is increasing, and people's energy in physical exercise is increasing [4]. Adequate physical exercise can maintain the health of bones and muscles, control body weight, reduce obesity, depression, and anxiety, and promote mental health [5]. Studies have shown that sports can improve college students' interpersonal relationship and psychological quality and promote college students' mental health.

When the material needs are initially met, people begin to pursue more spiritual life satisfaction, hoping to maintain a good mentality and harmonious interpersonal atmosphere. Therefore, people's demand for mental health services such as psychological counseling and psychotherapy is increasing [6]. Community health education refers to an organized, planned, and evaluated health education activity with the community as the unit, the community population as the object of education, and the goal of promoting the health of the community masses [7]. Health education and health promotion are activities to create a healthy environment, disseminate health-related information, improve people's health awareness and self-care ability, advocate healthy behaviors and lifestyles, and promote the improvement of people's health quality [8]. How to improve the health literacy of residents has gradually become the primary problem faced by public health organizations. The traditional health education mode is carried out through lectures or paper brochures, and the effect is not significant, so we need to constantly improve the health education mode. Community health education is particularly important in community mental health service.

Mental health is a sound state in which people have reasonable cognition, stable emotion, appropriate behavior, interpersonal harmony, and adapt to changes in the process of growth and development. Mental health service is to use the theories and methods of psychology and medicine to prevent or reduce various psychological and behavioral problems, promote mental health, and improve the quality of life, mainly including mental health publicity and education, psychological counseling, treatment of mental diseases, and psychological crisis intervention. Mental health is an important part of health, which is related to the happiness and well-being of the people and affects the harmonious development of society. Strengthening mental health services and improving the social psychological service system are the key measures to improve the public's mental health level, promote social psychological stability and interpersonal harmony, and enhance the public's sense of happiness. They are the basic requirements for cultivating good moral fashion, promoting coordinated economic and social development, cultivating and practicing the core values of socialism, and are a source of the country's long-term stability basic work.

## 2. The Basic Idea of Community Sports Public Service System Construction

At present, the urban community sports in China refers to the local mass sports, which is based on the natural environment and sports facilities in a certain area where people live together, with all community members as the main body, with the main purpose of meeting the sports needs of community members, enhancing the physical and mental health of community members, and consolidating and developing community feelings. As a planned, organized, and systematic social and educational activity, the core of health education is to encourage people to actively change unhealthy health behaviors and related factors affecting health behaviors, eliminate or reduce risk factors affecting health, master healthcare knowledge, establish health concept, prevent diseases, promote health, and improve quality of life. Urban community sports public service is an important concept to study social sports public management [9]. From the perspective of concept scope, the urban community sports public service system includes maintenance public service, economic public service, and social public service. Its scope is wider than other public services. Community sports is an important part of Chinese mass sports and the foundation of harmonious development of sports with Chinese characteristics. In practice, we should make full use of the advantages of community service function, carry out community service demand survey, understand the characteristics of population distribution, and gradually carry out mental health services suitable for community characteristics. Then, combined with the theory in the community practice, the standardized operation of community health education is formulated, and the standardized mode suitable for universal promotion is studied.

With the development of regional economy and society and the acceleration of urbanization, China's community sports public service system is in a critical period of construction and improvement. To establish a perfect community sports public service system is to provide more rich cultural life for community residents and provide conditions for residents to improve their physical quality. Community health service institutions should actively carry out professional training for full-time staff of community health education and strengthen the knowledge updating of health education staff such as general practitioners, nurses, and preventive healthcare personnel, as well as the skill training of health education, so as to improve the service quality of community health education [10]. The new public management theory mainly adopts the management method of entrepreneurs and improves the administrative performance by strengthening the market competition and guidance. This market efficiency oriented government reengineering movement ignores the democratic value and people's will. The construction of community sports service system has become an important issue of sports construction in the current social and economic transformation period, which is of great significance to promote the improvement of social life quality. The low efficiency or inefficiency of resource allocation caused by market limitations and defects cannot solve the problems of external economy and external diseconomy and social equity.

Health education can help to improve people's knowledge of chronic diseases and actively examine their own living habits and eating habits, so as to strengthen active prevention, reduce the occurrence of various chronic diseases, and improve the quality of life. As given in Table 1, it is a survey of the problems that need to be solved urgently in social sports.

The urban community sports public service system has the characteristics of sharing, nonprofit, and social benefits in the first place. The construction of the urban community sports public service system should focus on the development of urban community sports science and technology innovation services on the basis of daily sports facilities, sports organizations, sports guidance, and physical fitness testing. Fitness exercise can significantly regulate anxiety, depression, and other adverse emotional states and can produce good emotional effects, especially for those with mild and moderate anxieties and depression. The new public service theory puts citizens at the center of the whole governance system and pushes the spirit of public service, emphasizing that the role of government governance turns to service instead of steering and rowing, with the aim of enhancing the value of public service. People who exercise regularly can devote themselves to sports selflessly and generate interest and enjoyment directly from the activity process itself. At the same time, under the “encouragement” of such interest and enjoyment, it is beneficial to maintain their regular exercise.

## 3. The Basic Strategy of Perfecting the Construction of the Community Sports Public Service System

Without a sound community sports public service network, it is difficult to carry out community sports public service activities. Only a stable, high-quality professional backbone team, and consciously undertaking the functions of community sports, can we carry out community sports public service activities in an all-round, systematic, and long-term way. Social and economic formation is the basis and an important part of social formation. Economic transformation is the decisive factor of social transformation. With the increasing competition in modern society, people are under great psychological pressure from work, study, and life. In order to meet the needs of work, many people hide themselves and live with “masks,” which brings hidden dangers to their mental health [11]. Most of the community residents exercise with the nature of group; at the same time, because the fitness exercise is characterized by excitement and full of activities, the body and mind of the fitness exercise participants are in a certain degree of activation, through long-term, quantitative, regular fitness exercise, and can significantly improve the vitality of the body, which promotes the participants to better maintain interpersonal relationship.

The urban community sports public service system is the basic platform for the government to exercise social management functions and provide sports public services. It is an important guarantee for building a harmonious community and belongs to the category of public financial support. The evaluation of community sports public service often involves many factors or indicators. At this time, it is required to evaluate things according to multiple factors, but not according to the situation of a single factor. The structure of the community sports psychological prevention method system is shown in Figure 1.

Before solving the basic survival needs, people's livelihood issues are important, and it is understandable that sports investment ranks lower in public investment. With the progress of society and the increase of leisure time, people have changed their traditional leisure, which only pursues physical recovery and is limited to physiological self-cultivation, and started to change from recuperation to all-round development, with pleasure, relaxation, and health as the main purpose, and sports activities with positive and free subjective attitude have entered people's leisure life. With the improvement of living conditions, people's demand levels will continue to rise, and after meeting basic material consumption, they will pursue higher-level enjoyment needs and development needs. Public interest is not a simple aggregation of individual interests, but an agreement is reached through dialogue and consultation of public interests. Only by making the government aware of the importance of developing community sports construction can the related work be better implemented. Community sports have a wide environment, diverse contents, and flexible ways. Participants can choose their favorite sports freely and independently, which can enable participants to give full play to their abilities and cultivate their lively and cheerful personality.

Scientific and healthy community sports lifestyle pursues a healthy, active, and high-quality modern life goal. Through community physical exercise, the immune function of human body to diseases can be enhanced, the physical quality of human body can be improved, and the functional degradation of human body can be resisted. For example, Table 2 provides the estimation and significance test of structural parameters of China's social transformation indicators.

For psychological evaluation, whether to achieve the purpose of psychological evaluation is an important basis to measure the success or failure of work. The energy for a state can be defined as

(1) $$\begin{array}{c} w_{ij}=w_{ij}+a\left(\frac{X_{i}}{m}-w_{ij}\right). \end{array}$$

Adopt the bee colony optimization algorithm to deeply mine data and use quadratic correction function:

(2) $$\begin{array}{c} o_{k}=f\left(net_{k}\right)net_{k}=\sum_{j=0}^{m}w_{jk}y_{j}\\ y_{j}=f\left(net_{j}\right)net_{j}=\sum_{i=0}^{n}v_{ij}y_{j}. \end{array}$$

By being a polynomial kernel function,

(3) $$\begin{array}{c} E_{RME}=\sqrt{\frac{1}{P}\sum_{p=1}^{P}{\left(E_{P}\right)}^{2}}. \end{array}$$

Construct a parameter index distribution model of psychological evaluation with high-dimensional feature distribution space:

(4) $$\begin{array}{c} \Delta v_{ij}=\eta \delta_{j}^{y}x_{i}=\left(\sum_{k=1}^{l}\delta_{k}^{o}w_{jk}\right)\left(1-y_{j}\right)y_{j}x_{i}. \end{array}$$

Community sports is a sports activity integrating entertainment, leisure, and health. It has no fierce competition from competitive sports, can avoid the negative psychology caused by failure, and has no pressure to win or lose. All of it is decided by the sports themselves. In leisure time, the whole family can participate in community sports activities together, which can not only exercise and enrich the spiritual and cultural life of the family but also make the family understand each other, create common hobbies, increase the cohesion of the family, make the family harmonious and unite, and maintain social stability. The noumenon meaning of sports consumption is the personal consumption behavior of pursuing development and enjoyment after satisfying the basic living consumption, and it is also the personal consumption behavior of individuals in their spare time after completing normal work and necessary housework. At present, the competent departments of the community sports public service system at all levels are not clear, community sports organizations seldom adopt the way of community management, and there is no relationship between rights and obligations between communities and members [12]. The community sports organization management service system is one of the important means to mobilize residents to participate in fitness activities, which plays an important role in helping community residents achieve fitness goals and then achieve community sports work goals. The relationship between government and citizens is different from that between enterprises and customers. Public managers should not only respond to the needs of citizens but also pay more attention to cultivating the cooperative relationship between government and citizens.

## 4. Conclusions

Regular physical exercise can significantly enhance the adaptability of individuals, improve interpersonal relationships, eliminate psychological barriers, and play an important role in improving mood, keeping a good mood and promoting the healthy development of individual psychology. China's investment in social sports is far less than that in competitive sports in the same period. The lack of public investment is an important reason for the low level of mass sports and the weak awareness of mass sports. In order to achieve practical results, the government needs to issue relevant policies, organize and implement specific measures, and realize the balanced supply policy for the construction and development of the urban community sports public service system. Scientific and healthy community sports lifestyle pursues a healthy, active, and high-quality modern life goal. Through community physical exercise, the immune function of human body to diseases can be enhanced, the physical quality of human body can be improved, and the functional degradation of human body can be resisted. The community sports public service system is the top priority for the development of social sports work at present. Only clarifying the orientation and development direction of the community sports public service system can community sports public service achieve long-term and stable development.

## Figures and Tables

**Figure 1:** The system structure of community sports psychological prevention methods.

**Table 1:** Investigation on the urgent problems of social sports.

Urgent problems	Select headcount	Proportion (%)
Construction of sports facilities	7101	72.5
Organize sports activities regularly	4824	49.2
Establish various sports organizations	3772	38.5
Strengthen sports publicity and mobilization	2252	23.0
Sports skills training	2341	23.9
Others	355	3.6

**Table 2:** Information fusion parameter estimation and significance test.

Path description	Fusion parameters	Path coefficient
Learning ability	7.55	7.57
Promotion ability	6.09	6.15
Management ability	7.17	6.53

## Data Availability

The data used to support the findings of this study are included within the article.
